# Dynamic Collaboration Model of Production Network Based on Cloud Service Bus

**DOI:** 10.1155/2022/8149132

**Published:** 2022-07-12

**Authors:** Yuan Zhao, Shifeng Liu

**Affiliations:** School of Economics and Management, Beijing Jiaotong University, Beijing 100044, China

## Abstract

The IT system of manufacturing enterprises usually has many problems, such as complex industrial software, different development languages, diverse communication protocols, and complex operation environment. Cloud service bus (CSB) technology based on service model encapsulates various applications existing in enterprises by means of the integration of cloud service bus and micro services, which can realize the rapid cloud migration and deployment of heterogeneous industrial application software. Theoretically, after the production system is connected to CSB, it can be arranged arbitrarily by service choreography technology to produce any possible products. However, in the context of industrial Internet, the production system connected to CSB corresponds to the equipment, materials, personnel, and other resources on the production line one by one. These production nodes need to consider the production capacity and cost of production service nodes and the output value of the whole production network, and cannot be combined arbitrarily. Therefore, when integrating production service nodes, we should not only consider the technical integration, but also consider whether the production conditions support this integration. To solve the problem of production node integration in CSB, a dynamic collaboration model of production network based on cloud service bus is proposed in this paper. The model takes the capacity, cost, and production relationship of production nodes as constraints, and the overall efficiency of production network as the optimization goal. The model can calculate the new creation, modification, deletion, and other scheduling operations of production line services in real time and give the production plan with the highest resource utilization and the greatest value in the current production network. The model can improve the rationality and economy of service choreography and give full play to the value of production network. Taking an enterprise with 11 production nodes and 5 production lines as an example, this paper discusses in detail how to use this model to calculate the optimal production organization scheme and the maximum output value of the enterprise.

## 1. Introduction 

There are many problems in the IT system of manufacturing enterprises, such as complex industrial software, different development languages, diverse communication protocols, and complex operation environment. These software have great differences in connection form and management relationships. In the context of Industrial Internet, it is difficult for the production systems of these enterprises to access cloud computing. In view of the problems of various industrial communication protocols and complex operating environment of industrial software in manufacturing enterprises, CSB technology supports the service access, opening and conversion of multiple protocols, supports flexible and customized data transformation, supports the connection and integration of heterogeneous industrial software, and realizes the connectivity between enterprise organizations. CSB provides many adapter connectors, which can connect different types of applications and data services on local and cloud, effectively reducing the complexity of application system integration. The service choreography capability provided by CSB effectively solves the problems of choreography and unified application of heterogeneous industrial software after accessing the cloud level. At the same time, CSB uses the service choreography technology to combine and arrange multiple production service nodes according to the production process flow to form a production line. Multiple production lines interweave to form a production network. The production service node connected to CSB is mapped to the manufacturing resources on the production line. Therefore, any service choreography of production service nodes should consider the production capacity, cost, and other constraints of the actual production line. Only in this way can the production network realize the integration of online and offline and improve the efficiency of the whole production network.

The production capacity provided by the production node connected to the bus is scarce and limited. Moreover, enterprises pursue the maximization of overall interest when integrating production nodes. Therefore, how to optimize the overall efficiency of the production network under the condition of limited capacity and cost is the key problem to be solved in the research field of heterogeneous system integration. This paper introduces a dynamic collaboration model of production network based on CSB. This model applies complex network technology to systematically analyze the production network constructed by service scheduling technology, and puts forward a dynamic collaboration model of production node resources to maximize the overall efficiency of the production network under the condition of limited production node capacity. Based on the online and offline integration of node lines in CSB, the model makes decisions on whether the new production line can be arranged, and gives the maximum production scheme of the production network. This method can make full use of existing resources and dynamically optimize the production network.

The rest of this paper is organized as follows.  Section 2 reviews some related work, introduces the solution of CSB technology to integrate heterogeneous systems and analyses the problems faced by this solution in the actual production environment.  Section 3 investigates the heterogeneous system integration and service choreography based on CSB, and analyses the characteristics of industrial Internet using CSB integration.  Section 4 constructs a dynamic cooperative control model of production network based on CSB. In Section 5, through an example, this paper introduces how to apply the model to the dynamic cooperation of production resources to maximize the overall efficiency of the production network.  Section 6 concludes the whole paper.

## 2. Related Work

### 2.1. Heterogeneous System Integration

In the field of enterprise heterogeneous system integration, service-oriented architecture (SOA) is a common and mature method to solve enterprise heterogeneous system integration. Enterprise service bus (ESB) is the core component of SOA. It extends middleware by connecting heterogeneous components and systems and provides integration services. In addition, SOA also provides service choreography, service management, and other functions [1]. From the perspective of SOA architecture, it mainly solves the problems of heterogeneous system, technical access, and service quality management access. Service nodes in SOA mainly guarantee the quality of service through quality-of-service system (QoS), but QoS mainly manages the nonfunctional requirements of access services. The main evaluation indicators of QoS include response time, reliability, and availability.

### 2.2. Cloud Manufacturing

Cloud manufacturing is widely used in cross-enterprise integration in the manufacturing field. Based on the concept of manufacturing as a service, cloud manufacturing adopts new technologies such as cloud computing and Internet of Things to integrate the manufacturing resources connected to the network and provide high value-added, low-cost, and global product manufacturing services. Zhao et al. [2] combined with the characteristics of cloud manufacturing, discussed the connotation of manufacturing cloud service adaptation, including definition, characteristics, and content, and proposed a manufacturing cloud service adaptation technology framework composed of data source layer, data perception layer, data analysis and decision-making layer, and action execution layer. Xu et al. [3] proposed an adaptive bat algorithm (Saba) to solve the problem that optimizing and selecting appropriate services to complete manufacturing tasks is manufacturing services. Yin et al. [4] established a multi-agent-based manufacturing resource cloud service encapsulation adapter for the needs of distributed, heterogeneous and different conditions of manufacturing resource service encapsulation, and studied the adapter knowledge representation and accumulation method based on semantic directed graph.

### 2.3. Cloud Manufacturing Service Collaboration Based on Service Choreography

At present, many scholars have studied manufacturing service collaboration based on service choreography technology. Through the orderly choreography of different services connected to cloud services, the efficiency of cloud manufacturing service system can be effectively improved. Maythaisong and Songpan [5] proposed mutation-based harmony search algorithm to select web services and to compose with minimum defects. This algorithm can help find appropriate solutions to compose services based on business plans. Yin et al. [6] proposed a cloud manufacturing service scheduling method based on WS-CDL. By realizing the standardized description of cloud manufacturing service collaboration, it promotes the effective communication between cross-organizational services and achieves the purpose of improving the resource utilization of service providers. Kopp and Leymann [7] proposed a modelling choreography method based on WS-BPEL to solve the problem that there is no agreed standard to describe choreography. You [8] constructed the technical framework of service-oriented composition evolution method for large-grained web services and proposed the determination method of evolution type and influence scope for large-grained web service composition. Ojstersek and Buchmeister [9] and Grznar et al. [10] applied simulation technology to study the production optimization strategy of enterprises under resource constraints. Hwang et al. [11] studied the performance monitoring of message server and system based on MQTT. One of the core functions of CSB is to realize the message transmission between components stably and with low delay.

### 2.4. The Application of Complex System Theory

After the production service node is connected to CSB or cloud manufacturing system, it forms an intertwined mesh production system through service choreography, showing the characteristics of the complex network. Pan et al. [12] proposed a feasible architecture of multi-agent manufacturing system in a discrete manufacturing workshop to solve the problem of order uncertainty caused by the increase of customer personalized demand. Huang et al. [13] proposed a real-time dynamic scheduling mechanism of manufacturing system based on event triggering from the aspects of scheduling method, multi-agent coordinated control, and scheduling control algorithm. Li et al. [14] studied the multi-objective planning using ant colony algorithm, and verified through engineering practice that the optimized ant colony algorithm can avoid the low efficiency of optimal solution search and the shortage of initial pheromone.

To sum up, the research on heterogeneous system integration in the context of Industrial Internet mainly focuses on the following three aspects: firstly, SOA and cloud manufacturing technologies are used to solve the access integration problem at the technical level of heterogeneous services. Secondly, service choreography is used to solve the composition problem of discrete services. Finally, QoS is used to solve the quality assurance problem of access service. At present, there are few studies on the capacity of the connected production service node and the overall optimization of the production network.

## 3. Heterogeneous System Integration and Service Choreography Based on CSB

### 3.1. Heterogeneous System Integration Based on CSB

CSB technology realizes the encapsulation of heterogeneous systems through service encapsulation technology. Based on multi-protocol connection adaptation technology, CSB realizes the integration, choreography, governance, and other operations of heterogeneous systems, and finally provides services for internal and external applications of enterprises through a unified service gateway. The structure of CSB is shown in Figure 1:

In Figure 1, internal industrial software and external industrial software represent the internal and external software systems used by the enterprise in production. The function of service-oriented encapsulation component is to combine different types of production software into standardized service modules in a technical way. The multi-protocol adaptation gateway component is mainly used to adapt the industrial software with different communication protocols, so that the software with different communication protocols can communicate with each other.

To solve the problems of poor compatibility and inconsistent architecture of industrial software in manufacturing enterprises, CSB provides a unified and highly compatible heterogeneous software packaging solution to realize the service-oriented packaging of enterprise heterogeneous software. In view of the problems of diverse communication protocols and complex operating environment of industrial software in manufacturing enterprises, CSB provides multi-protocol adaptation gateway to support the service access, opening and conversion of common protocols, and flexible and customized data transformation, to support the connection and integration of heterogeneous industrial software and realize the connectivity between enterprise organizations. At the same time, CSB provides rich adapter connectors, which can connect different types of applications and data services on local and cloud, effectively reducing the complexity of application system integration. After accessing CSB, the service quality of production service nodes is guaranteed by QoS system. QoS can provide quality assurance for nodes, including reliability and response speed.

### 3.2. CSB-Based Service Choreography

After the heterogeneous software is connected to the service, it is managed by the service management function provided by CSB. The service choreography function provided by CSB will connect multiple production nodes of CSB, effectively, integrate the business process according to the operation process of product production, realize the reasonable choreography of various services, and form a new production line. In this way, enterprises can reuse existing heterogeneous assets, quickly solve the production problems of new products, reduce the cost of production line construction, and improve the ability of enterprise applications to market changes. The production node connected to CSB will be called by multiple production processes, and the processes of multiple production lines will be intertwined to form a complex production network system. The structure of the production network is shown in Figure 2.

As shown in Figure 2, the production line pool is the collection of all production nodes connected to the CBS. Service node pool is the collection of production control systems integrated into the system through CBS. The production line in the production line pool is the production line formed by the process engine connecting and combining multiple production nodes according to the product production scheme. Multiple production nodes and multiple production lines call and interweave each other to form a complex production network.

### 3.3. Characteristics of Industrial Internet Using CSB Integration

Under the condition of Industrial Internet, there is a big difference between the integration of heterogeneous systems using CSB and the integration that only provides computing, storage, and other services. The main differences are as follows:

1. Strong mapping relationship between online production nodes and offline production resources. Since the production nodes connected to CSB have a unique mapping relationship with the offline production system and resources, the reorganization of the offline production line corresponding to the assembly of online services needs to consider various factors, such as production capacity, cost, effective utilization of production resources, and maximization of the value of production products. This strong correspondence between online and offline resources has more restrictions on service integration under the CSB mode.
2. Production nodes are limited by many factors. Each production node has various resource constraints such as capacity and cost. Since each node corresponds to a unique production resource one by one, the capacity constraints of each node need to be considered. Therefore, production nodes cannot be accessed without restrictions.
3. The choreography of the production line is related to the production decision of the enterprise. Since the production line in CSB is the mapping of physical production lines, the profit of the enterprise should be considered in the combination of online production services and the production plan of each production line. To achieve the optimal efficiency of the production network, it is necessary to calculate and dynamically adjust the production strategy of products in the production network in real time, make full use of production resources, and maximize the profits of enterprises.

At present, there is no restriction strategy for production nodes in the cloud service integration architecture, and there is no strategy to achieve the optimal efficiency of the production line. Therefore, this paper proposes a dynamic collaboration model of production network based on CSB, which mainly solves the problems of service choreography and production planning after heterogeneous systems are connected to CSB. On the basis of fully considering the production constraints, the optimal combination of service choreography and production strategy is realized.

## 4. Dynamic Cooperative Control Model of Production Network Based on CSB

### 4.1. Structure of the Model

To realize the dynamic system control of production network, it is necessary to redesign the structure of the original production network and add the dynamic collaboration model. Based on the production network structure of CSB shown in Figure 2, the model is upgraded, and the structure is shown in Figure 3.

As shown in Figure 3, the function of the “Dynamic collaboration model” component is to dynamically control the service orchestration according to certain rules to ensure the availability and rationality of the production line. After the production control model is added to the production network, the operation of the service choreography engine can be controlled according to the agreed rules. The dynamic collaboration model of production network is an event-driven model, which can respond to the change events of the production network and realize the dynamic collaboration control of the production network, to achieve the optimal configuration of the network.

The operation mode of the collaborative control model is that the event processing center processes the events generated by the production node, production line, and production network according to the predefined processing rules and optimization objectives, and outputs the overall control strategy of the model. Its structure is shown in Figure 4.

As shown in Figure 4, the dynamic cooperative control model adopts the classical event processing model to realize the dynamic cooperative control. Event sources include: production node events, production line events, and production network events. Node events include production node addition, removal, capacity change, and cost change. Production line events include changes in the arrangement of production nodes, changes in product prices, and changes in the production priority of the production line. Production network events include changes in optimization objectives and restrictions. After the model change event occurs, it will be propagated to the registered listeners. The listener then passes the event to the event processing model for processing and outputs the control strategy. The control strategy mainly includes the change decision of nodes and production lines and production planning strategy.

### 4.2. Dynamic Collaborative Control Model of Production Network

This paper analyzes the network structure of heterogeneous systems based on CSB by using the theory and method of complex network systems.

According to the network structure in Figure 3, the production network is composed of production nodes and production line nodes. The production node represents the system that can provide production services connected to the CSB. The production line node is composed of the production line generated by the service node through choreography. Products need to be produced in a certain order, so the edges between nodes are directed. Edge connection indicates that there is a production combination relationship between nodes. Because the production of each product needs to consume the resources of the node, so each edge has a weight.

Let *G* be an abstract representation of the production network based on CSB, and define *G*(*S*, *P*, *E*, *W*) as a directed and weighted network, where: *S*={*s*_1_, *s*_2_, *s*_3_,…, *s*_*m*_}, *S* represents the collection of all production systems connected to CSB, *m* is the total number of production nodes connected in CSB, and each *s*_*i*_ represents the production resources responsible for completing certain business functions; *P*={*p*_1_, *p*_2_, *p*,…, *p*_*n*_}, *P* represents the set of production line nodes. Each production line is composed of multiple production service nodes according to a certain production order; *E*={*e*_1_, *e*_2_, *e*_3_,…, *e*_*l*_}, (*s*_1_, *s*_2_) ∈ *E*, *E* represents the set of production relations between production nodes, the directed edge of nodes *s*_1_ to *s*_2_ in the network, and the production dependency of *s*_1_ to *s*_2_ in the production process. Since the same node can be combined into multiple production lines, there are multiple edges derived from a specific node; *W*={*w*_1_, *w*_2_, *w*_3_,…, *w*_*k*_}, *W* is a set describing the weight of each edge. *w* means that the production of a specific product *p* needs to consume the capacity of the corresponding production node.

There are multiple production lines in production network *G*(*S*, *P*, *E*, *W*). The quantity and price of products produced by each production line are different, so the output value of production network *G* in unit time can be defined as:

(1) $$\begin{array}{c} V=\sum_{i=1}^{n}q_{i}\times v_{i}, \end{array}$$

where *V* represents the total output value of the production network, *n* represents the number of production lines, and *q*_*i*_ and *v*_*i*_ represent the output and price of line *p*_*i*_.

In the same way, the cost, consumption, and profit calculation functions of the production network can be defined. According to these functions, the optimization objectives of the model, such as maximum output value, maximum profit, and minimum cost, can be defined.

The constraints of the model mainly include node capacity, cost, and industrial logic requirements of upstream and downstream nodes. Next, the node capacity constraints are analyzed. In production network *G*, multiple production lines can share the same production node, that is, the same production node can provide services for multiple production lines. Let *O*_*s*_*j*__ represent the production capacity of node *s*_*j*_, and *w*_*p*_*i*_*s*_*j*__ represent that the production line *p*_*i*_ needs to consume the production capacity of production node *s*_*j*_. In the production network, the capacity consumed by any production line using the same production node cannot exceed the capacity of that node. This relationship can be defined as:

(2) $$\begin{array}{c} \sum_{i=1}^{n}w_{p_{i}s_{j}}\leq O_{s_{j}}. \end{array}$$

Based on the above analysis, the optimal production plan of production network *G* can be described as the optimal production plan to realize the output value, cost, and profit of production network under the constraints of capacity and cost of each node. If the maximum output value is taken as the optimization objective, the objective function of the model is as follows:

(3) $$\begin{array}{c} \max\left(V\right)=\max\left(\sum_{i=1}^{n}q_{i}\times v_{i}\right). \end{array}$$

There are two main factors that affect the decision-making of an enterprise. First of all, the production line arrangement affects the product category decision of the enterprise. The products produced by different production lines bring different profits to the enterprise, so the enterprise needs to make decisions on which production lines to arrange. Second, the production line arrangement affects the output decision of each production line. Because production lines need to consume the capacity of production nodes, enterprises need to make decisions on the output of each production line under the condition of limited capacity.

According to the business needs of the enterprise, the user can establish the set of constraints in the way of equation (2), establish the optimization objective function according to the requirements of equation (3), and finally form the optimization control model.

### 4.3. Application of the Production Network Dynamic Collaboration Model

Combined with the service choreography capability provided by CSB, the production network dynamic collaboration model can realize the following functions:

1. Dynamic control of production nodes. After the production node is changed, the model realizes resource control and early warning by monitoring whether the resources of the production node are within the limit.
2. Dynamic capacity expansion and adjustment of production nodes. The model can calculate the resource consumption of production network nodes in real time, and enterprises can find the bottleneck nodes. Enterprises usually face the decision of expanding production nodes. Combined with the decision-making objectives of the model, the model can calculate the costs and benefits of capacity expansion nodes and provide a basis for enterprises to make capacity expansion decisions.
3. Dynamic control of production line editing. Managers need to judge the impact of these operations on the production line and the whole network when adding, modifying, and deleting the production line. This model evaluates the impact of production line changes on the overall income of the enterprise by calculating the income of the production line itself and the network, and provides decision-making basis for managers.
4. Dynamic adjustment of production strategy. In the production network, if the production capacity and price of products change, and the optimal target rules of the model are adjusted, the model can control which production lines are produced and how many are produced.

## 5. Model Validation and Application

In the context of Industrial Internet, production enterprises can use the heterogeneous system integration, service management, service choreography, service control, and other functions provided by CSB to carry out the flexible combination of production lines according to the market demand, to realize the rapid integration of internal and external resources of enterprises.

Taking a production enterprise as an example, this part explains the operation mechanism of the production network dynamic collaboration model based on CSB through the control of nodes, production lines, and networks. There are 11 internal and external production nodes integrated by the enterprise, which are combined into 5 production lines through the service choreography group function provided by CSB. The structure of the production service nodes included in the five production lines is shown in formula (1).

(4) $$\begin{array}{c} P=\left[\begin{array}{c} p_{1}\left(S_{1},S_{2},S_{3},S_{4},S_{5}\right)\\ p_{2}\left(S_{1},S_{2},S_{3},S_{4},S_{6}\right)\\ p_{3}\left(S_{7},S_{8},S_{9}\right)\\ p_{4}\left(S_{1},S_{2},S_{7},S_{10}\right)\\ p_{5}\left(S_{3},S_{8},S_{11}\right) \end{array}\right]. \end{array}$$

The value of the production line in the production network can be expressed as: *V*={*v*_1_, *v*_2_, *v*_3_, *v*_4_, *v*_5_} where *v*_*i*_ is the value generated by the production line *p*_*i*_.

According to the characteristics that the production network *G* conforms to the bisection network [15], the projection method is used to analyse the production network *G*, and the structure diagram of the production network can be obtained, as shown in Figure 5.

In Figure 5, there are 11 nodes, 15 interactive edges, and 5 production lines to produce 5 different products. The price of each product is different. Since the same production node can serve multiple production lines, there are multiple edges between two production nodes. The weight *w*_*p*_*k*_*i*_ on each edge indicates that production line *p*_*k*_ needs to consume the capacity of production node *S*_*i*_. The weight matrix of the production network is as follows:

(5) $$\begin{array}{c} w=\left[\begin{array}{c} w_{1}\left(w_{p_{1}1},w_{p_{1}2},w_{p_{1}3},w_{p_{1}4},w_{p_{1}5}\right)\\ w_{2}\left(w_{p_{2}1},w_{p_{2}2},w_{p_{2}3},w_{p_{2}4},w_{p_{2}6}\right)\\ w_{3}\left(w_{p_{3}7},w_{p_{3}8},w_{p_{3}9}\right)\\ w_{4}\left(w_{p_{4}1},w_{p_{4}2},w_{p_{4}7},w_{p_{4}10}\right)\\ w_{5}\left(w_{p_{5}3},w_{p_{5}8},w_{p_{5}11}\right) \end{array}\right]. \end{array}$$

The dynamic collaboration model of production network proposed in this paper aims at maximizing the output value of the production network. According to the above analysis, the optimal production function of this enterprise can be expressed as:

(6) $$\begin{array}{c} \text{Max}\left(p\right)=V*Q, \end{array}$$

where *V* is the value set of each product, and *Q* is the quantity produced by each production line. One production node can be used by multiple production nodes. The total capacity of a node consumed by multiple production lines cannot exceed the total capacity of the node. The capacity of any production node *S*_*i*_ should meet the conditions expressed in formula (2).

The production node capacity, consumption of each production line, and product price of the production enterprise are shown in Table 1.

By substituting the data in Table 1 into formula (6) the production dynamic control model of the enterprise can be obtained. This paper uses the linear programming method of operations research to solve it. The results of model calculation are shown in Tables 2 and 3.

Because the production data in Table 1 corresponds to the nodes and edges of the production network in Figure 5, the changes of the network model will be transferred to the model parameters. This change triggers the calculation of the model through the event transmission mechanism to realize the purpose of dynamic collaborative control of network change. Managers can make decisions based on the results calculated by the model. The specific applications of the model are shown as follows.

1. Real-time calculation of the optimal production plan of the production network. Bring the production data in Table 1 into formula (2) and use the linear programming method of operational research to find that when the product output *q*={11,8,9,0,1}, *v*={1430,840,1800,0,130}, the maximum output of the production network can be 4200 under the condition of meeting the constraints of the production node.
2. Collaborative analysis of production node capacity. The model can calculate the capacity consumption of each production node when the output value of the production network is maximized. Managers can make scientific decisions according to the capacity consumption of production nodes. For example, it can be seen from the calculation results that the consumption of production node *S*4 is close to the production capacity. This may be a key node restricting the capacity of the entire production network. For nodes with large capacity surplus, enterprise managers can fully consume the remaining capacity by developing new products, or share the capacity on the Industrial Internet to realize cross-organizational capacity optimization; for production nodes that tend to be saturated with capacity, enterprise managers can expand the capacity of nodes to expand production and increase enterprise income.
3. Collaborative decision analysis of production line. The model can provide decision support for the change of production line. It can be seen from the calculation results that the output of *P*4 is 0, that is, no production is carried out. The manager can decide whether to remove production line P4. Furthermore, if the maximum output value of the production network is reduced after the new production line is added, the production line cannot join the production network. Otherwise, you can join the production network. In production practice, it is necessary to realize the optimization of production network under the condition of product output limitation. The model proposed in this paper also supports this scenario and only needs to add the output limit condition of the production line to the limit condition of the model.

## 6. Conclusion

Manufacturing enterprises use the Industrial Internet to realize cross-organizational business integration. The enterprise encapsulates the existing capacity into services and deploys them in the cloud service environment. With the integration capability provided by CSB, the integration of internal and external production services is realized to meet the requirements of flexible production and intelligent manufacturing. In this paper, we systematically introduce the technical system of production service integration and choreography based on CSB, and propose a dynamic collaboration model of production network based on CSB. Then, we use the theory and method of complex network to model the production network based on CSB, and establish a dynamic collaboration model, which provides support for the realization of dynamic collaboration control of service choreography. Finally, an example is used to introduce the application method and effect of the model in detail.

By adding the dynamic collaboration model to CSB system, this paper solves the problem of dynamic collaboration control in CSB model and improves the rationality and economy of production network. In the process of model building, this paper does not consider the time consumed by the node to produce unit products, which may lead to the production line unable to produce as planned. Next, we will do further research in application scenarios such as multi-factor constraints and multiobjective collaboration to optimize the model and improve the generalization ability of the model.

## Figures and Tables

**Figure 1:** Structure of CSB.

**Figure 2:** Structure of the production network.

**Figure 3:** Service choreography and control model.

**Figure 4:** Dynamic cooperative control model based on event processing.

**Figure 5:** Production network diagram.

**Table 1:** Production information of network.

Category	*P*1	*P*2	*P*3	*P*4	*P*5	Capacity
*S*1	16.8	30.4	0	25.3	0	800
*S*2	15.9	25.4	0	29.3	0	400
*S*3	30.5	0	0	0	40.2	500
*S*4	42.3	15.6	0	0	0	600
*S*5	22.1	0	0	0	0	700
*S*6	0	20.3	0	0	0	500
*S*7	0	0	32	16.3	0	300
*S*8	0	0	24.3	0	20.5	250
*S*9	0	0	33.4	0	0	350
*S*10	0	0	0	25.5	0	300
*S*11	0	0	0	0	39.5	350
Price	130	105	200	155	130	—

**Table 2:** Consumption of production node capacity.

Category	*S*1	*S*2	*S*3	*S*4	*S*5	*S*6	*S*7	*S*8	*S*9	*S*10	*S*11
Capacity	800	400	500	600	700	500	300	250	350	300	350
Consumption	428	378.1	375.7	590.1	243.1	162.4	288	239.2	300.6	0	39.5

**Table 3:** Output and output value of production line.

Category	*P*1	*P*2	*P*3	*P*4	*P*5
Price	130	105	200	155	130
Quantity	11	8	9	0	1
Value	1430	840	1800	0	130

## Data Availability

The data used to support the findings of this study are included within the article.
